# An Inhibitor of Nuclear Factor-Kappa B Pathway Attenuates the Release of TGF-*β*1 and Inhibits the Fibrogenic Progress in a Model of Airway Remodeling Induced by Acrolein

**DOI:** 10.1155/2022/4984634

**Published:** 2022-04-06

**Authors:** Peng Chen, Xiaoxia Wang, Yanping Li, Hong Liu

**Affiliations:** ^1^Department of Respiratory Medicine, The Third People Hospital of Chengdu, Chengdu, Sichuan 610031, China; ^2^Department of Radiology, The Third People Hospital of Chengdu, Chengdu, Sichuan 610031, China

## Abstract

Airway inflammation, airway hypersecretion, and airway remodeling are believed to be involved in the process of lung fibrosis. Nowadays, acrolein is widely used to establish the model of airway remodeling. An active component of propolis, named caffeic acid phenethyl ester (CAPE), is recognized as an inhibitor of the NF-*κ*B pathway and shows anti-inflammatory effect. The purpose of this study was to investigate the protective effect of CAPE on acrolein-induced airway remodeling. 24 mice were divided into 4 groups: control group; acrolein group, mice received acrolein (inhalation of acrolein for 20 days); CAPE group, mice received CAPE (30 mg/kg); and acrolein+CAPE group, mice received acrolein and CAPE. After 20 days, lung tissue was removed for histopathology and immunohistochemical evaluations. TGF-*β*1 and Muc5ac levels were measured at the protein and molecular levels. Additionally, the phospho-P65/P65 values in the airway smooth muscle cells treated with TGF-*β*1 or CAPE were detected by Western blot. The results showed that compared with the control, subepithelial collagen deposition, airway inflammation, and peribronchus fibrosis were inhibited in the group treated with CAPE. Furthermore, TGF-*β*1 was significantly decreased in the acrolein+CAPE group compared with the acrolein group. Additionally, we identified CAPE inhibited P65 phosphorylation. However, CAPE did not inhibit the Muc5ac overproduction and hypersecretion induced by acrolein. In conclusion, as an inhibitor of the NF-*κ*B pathway, CAPE attenuated the release of TGF-*β*1_,_ which inhibited the fibrogenic progress induced by acrolein in mice and took no effect on inhibiting airway mucus hypersecretion.

## 1. Introduction

Repeatedly airway inflammatory injury, imperfect tissue repair, and aberrant fibrosis are now recognized as key pathophysiological features of inflammatory diseases of the airways, including cystic fibrosis, bronchiectasis, and chronic obstructive pulmonary disease (COPD). Airway inflammation, airway hypersecretion, and airway remodeling are believed to be involved in the process of pulmonary fibrosis (PF) [1–3]. Nowadays, the underlying mechanisms involved in lung fibrosis remain obscure and conventional therapeutic strategies, including glucocorticoid and oxidation inhibitor, have limited efficacy in treating PF [4]. Therefore, we tried to find more effective drugs for the treatment of PF.

In the last decade, many studies have revealed that some particular cellular signaling pathways have been involved in such fibrogenic process [5, 6]. In animal experiments [7, 8] and in vitro [9], blocking cellular signaling pathway at different stages may inhibit the fibrogenic process to some extent at least. The nuclear factor- (NF-) kappa B (NF-*κ*B) signaling pathway not only participates in cell growth and differentiation but also takes part in the inflammation reactions by regulating the expression of related genes, which is related to the fibrogenic progress [10, 11]. P65 is an important member of the NF-*κ*B family. The phosphorylation of P65 initials the activation of the NF-*κ*B pathway. Transforming growth factor beta (TGF-*β*) is a factor synthesized in a wide variety of tissues, which is believed to play an important role in cellular differentiation, embryonal development, immune function, and hormone secretion [12]. TGF-*β* is found mostly as homodimer forms of separate gene products TGF-*β*1, TGF-*β*2, or TGF-*β*3. Currently, TGF-*β*1 has been found to induce NF-*κ*B p65 phosphorylation and mediate collagen synthesis [13]. Verma et al. [14] also discovered that quercetin-3-rutinoside attenuates radiation-induced lung inflammation and fibrosis by modulating the NF-*κ*B/TGF-*β*1 signaling pathway.

A low-molecular-weight aldehyde found in photochemical smog and tobacco smoke, named acrolein, can induce mucus hypersecretion, airway inflammation, and airway remodeling [15, 16]. Acrolein-induced mucus hypersecretion is accompanied by mucous cell differentiation and followed by fibrogenic process, which may be related to the pathogenesis of cystic fibrosis, bronchiectasis, and COPD. Recently, acrolein has been widely used to establish the model of airway remodeling [17, 18]. However, the fibrogenic phenotype and the increased level of TGF-*β*1 induced by acrolein have not been fully reported in the mice model.

Caffeic acid phenethyl ester (CAPE) is an active component of honeybee propolis. In recent years, CAPE has been recognized as a phenolic antioxidant and is known to have potential anticancer, anti-inflammatory, antimicrobial, and other beneficial medical properties [19, 20]. The underlying mechanisms refer to the suppression of NOX4 expression [21], inhibition of the MAPK/NF-*κ*B signaling pathway [22], and so on. Through inhibition of NF-*κ*B signaling, CAPE had a protective effect *in vitro* [23] or in amiodarone-induced PF rat model [19]. However, the potential property of antifibrosis of CAPE has not been observed in an airway remodeling process induced by acrolein in mice.

Mucus overproduction and hypersecretion are also involved in the process of airway remodeling [24]. Mucin 5AC (Muc5ac) is a representative mucus protein [25]. Cheng et al. showed that microRNA-145 decreased Muc5ac expression to attenuate airway remodeling [26]. Therefore, based on the above study, in the current study, we investigated the fibrogenic progress in mice treated with acrolein inhalation, evaluated the dynamic changes of TGF-*β*1 and Muc5ac level, and tested the interventional effect of CAPE.

## 2. Materials and Methods

### 2.1. Animals

The Animal Care and Use Committee of West China Hospital of Sichuan University approved this animal study. Specific pathogen-free (SPF) grade male C57BL/6 mice (20~30 g) (National Rodent Laboratory Animal Resources, Shanghai Branch, Shanghai, China) at the age of 4 weeks were used for experiments. The mice were housed in independent chambers (0.7 m × 0.4 m × 0.6 m, equipped with ventilation holes) and were maintained on a 12 h diurnal cycle with water and food provided ad libitum. Each chamber was at a temperature of 23 ± 3°C with a relative humidity of 50 ± 5%.

Consulting the animal model of mucus hypersecretion made by Ying et al. [27], we established an airway remodeling model induced by acrolein in mice. 24 mice were randomly divided into 4 groups (*n* = 6 for each group): control group, no treatment; acrolein group, mice received acrolein (inhalation of 0.0004% acrolein fog 6 h a day on 20 consecutive days in a chamber); CAPE group, mice received CAPE (30 mg/kg) via intraperitoneal injection every other day, and acrolein+CAPE group, mice received acrolein and CAPE.

### 2.2. Tissue Preparation

On the 20^th^ day, each mouse was anesthetized by intraperitoneal injection with 2% pentobarbital sodium before tissue collection. The chests were opened, and the lungs were excised completely, which were carefully washed off the bronchoalveolar lavage fluid (BALF) and fixed by 4% paraformaldehyde subsequently. After being embedded in paraffin, tissue sections were reserved for hematoxylin-eosin (H&E) and Masson stains.

### 2.3. BALF Collection

BALF was collected through a tracheal cannula with physiological saline on day 20 after anesthesia. Physiological saline (1 ml) was used to inflate the lung, and the lavage fluid was recovered with 90% of the original volume, which was reserved for total cell count. The lavage fluid was centrifuged at 400 × g for 15 min at 4°C. The cell-free supernatant was kept at a temperature of -70°C, while the sediment was prepared for differential cell count under a microscope.

### 2.4. Histopathology

Tissue sections were reserved for H&E stain to observe the morphologic changes of airway and peribronchus including mucus hypersecretion, infiltration of inflammatory cells, and proliferation of alveolar epithelial cells. Masson stain was made to evaluate the degrees of subepithelial collagen deposition and peribronchus fibrosis. The images were analyzed with Image-Pro plus 4.5 Software (Media Cybernetics Co, USA). And based on that, each sample's Ashcroft score was recorded according to the average scores from different visual fields under a light microscope [28]. This score was operated by four observers.

Hydroxyproline concentration of lung tissue was detected by a hydroxyproline assay kit (Nanjing Jiancheng Bioengineering Institute, Nanjing, China) in accordance with the manufacturer's protocol.

### 2.5. Enzyme-Linked Immunosorbent Assay (ELISA)

Total protein in BALF was evaluated using the Bradford method. TGF-*β*1 and Muc5ac protein levels in BALF were determined according to the instruction of the commercial ELISA kits (OriGene, USA). Samples were measured photometrically by an automated plate reader.

### 2.6. Reverse Transcription-Quantitative Polymerase Chain Reaction (RT-qPCR)

Total RNA was extracted from pulmonary tissue homogenates with TRIzol (Invitrogen Co., USA) and reverse transcribed, and then, the complementary DNA was amplified by polymerase chain reaction with the PCR kit (Takara Bio Inc., Dalian, China). Primers are as follows: forward, 5′-CAGCCTATGTGAAAGATGCC-3′ reverse 5′-GTAGAGGGAAGTGGAGTTATTGC-3′ for Muc5ac and forward 5′-TGTCACCAACTGGGACGATA-3′ reverse 5′-AGGTCTTTACGGATGTCAACG-3′ for *β*-actin. The products amplified were separated by agarose gel electrophoresis and visualized by Bio-Rad system. Relative quantity of Muc5ac mRNA was obtained by a comparative method using *β*-actin as an internal control.

### 2.7. Western Blot

Airway smooth muscle cells were obtained from normal airways of mice by tissue isolation. This experiment was divided into 3 groups: (a) blank control group; (b) TGF-*β*1 group, the smooth muscle cell was treated with 10 ng/ml TGF-*β*1 for 30 minutes; (c) TGF-*β*1+CAPE group, before stimulation with TGF-*β*1, the cell was pretreated with CAPE (100 nM) for 30 minutes.

After that, whole-cell lysate was extracted and antibodies against P65 and phospho-P65 (p-P65) (Cell Signaling Technology, USA) were used for immunoblot. The results were expressed by histogram which was based on the values of p-P65(p-P65)/P65 from 3 independent experiments.

### 2.8. Statistical Analysis

Statistical analysis was performed with SPSS 22.0 software. Data was expressed as mean ± standard deviation (SD). The comparisons between each group were analyzed by *t*-test. *P* values < 0.05 were considered significant.

## 3. Results

### 3.1. General Condition

Mice in the acrolein group and acrolein+CAPE group developed lassitude and anepithymia after inhalation of acrolein fog for 1 week. And 20 days later, the mice became languid and unresponsive as well as their furs turned matt. Moreover, the mice lost weight compared with the control and acrolein groups.

### 3.2. Morphological Changes

Compared with the control group, obvious mucus hypersecretion, mass infiltration of inflammatory cells, serous effusion, and proliferation of alveolar epithelial cells were observed in airway and peribronchus tissues of mice in the acrolein group (Figure 1(a)). Some alveolar epithelial cells thicken as the shock induced by acrolein progresses. What is more, we discovered fibrosis of peribronchus tissue, which was visually hyperplastic and septus. All these results above were evaluated by Ashcroft score (Figure 1(b)). The Ashcroft score was significantly higher in the acrolein group compared to the control group. However, CAPE treatment significantly reduced the scores of rats in the acrolein group.

Further by Masson staining (Figure 2), we found that the lung tissue of mice in the acrolein group showed significant collagen deposition, airway interval thickening, and peribronchus fibrosis. However, after CAPE treatment, the collagen fibers were reduced. These results suggested a potential protective effect of CAPE on such a pathological process.

### 3.3. Total and Differential Cell Count

After inhalation of acrolein for 20 days, mucus overproduction and increased serous effusion as well as infiltration of inflammatory cells were noticed in the mice. Total cell count and neutrophilic granulocyte count in the acrolein group were significantly increased in BALF compared with the control group (*P* < 0.05), which were evidently reduced after the treatment with CAPE (*P* < 0.05, compared with the acrolein group) (Figure 3).

### 3.4. Hydroxyproline Concentration of Lung Tissues

Hydroxyproline concentration of lung tissue was an indicator of the change of the collagen fiber level. There was no statistical difference between each group (*P* > 0.05) (Figure 4).

### 3.5. TGF-*β*1 Level in BALF

After collecting BALF from each group of mice, we measured the level of TGF-*β*1 by ELISA. TGF-*β*1 level in BALF was visually increased after inhalation of acrolein for 20 days (*P* < 0.05, compared with the control group), which was significantly reduced through intraperitoneal injection with CAPE (*P* < 0.05) (Figure 5).

### 3.6. Muc5ac mRNA and Muc5ac Protein Levels

By RT-qPCR and ELISA, we observed visible increases of Muc5ac mRNA level in lung tissue and Muc5ac protein in BALF after treated with acrolein (*P* < 0.05, compared with the control group). However, the increased levels of Muc5ac mRNA and muc5ac protein were not affected by the administration of CAPE (Figures 6 and 7). This suggested the inhibitions of airway mucin overproduction and hypersecretion were not the roles that CAPE played.

### 3.7. P65 Phosphorylation

After stimulated with TGF-*β*1, phospho-P65 level was increased in the airway smooth muscle cells. However, the expression was reversed by pretreatment with CAPE (*P* < 0.05) (Figure 8), which suggested the inhibition effect of CAPE on P65 phosphorylation induced by TGF-*β*1.

## 4. Discussion

Airway remodeling is characterized by proliferation of smooth muscle cells and deposition of extracellular matrix, which narrows the airway and enhances the bronchial hyperresponsiveness. Together with airway inflammation and airway hypersecretion, airway remodeling is believed to be involved in the process of PF [1, 2]. Smoking inhibits the immune response of T cell in pulmonary and disorders the tissue repair, which causes complex pathological progress as above. For a long time, it has remained obscure what has been the crucial component of cigarettes to play such a role. Lambert et al. declared acrolein, a kind of aldehydes extracted from cigarettes, inhibited T cell response and was related to the NF-*κ*B signaling pathway by alkylating cysteine and arginine residues [29].

As we know, the pathologic process of interstitial lung disease is commonly divided into two phases: inflammatory phase and fibrosis phase. Nowadays, many kinds of animal models are used to reproduce this process. Some researchers believe the “switch” between inflammation and fibrosis appears to occur around day 9 after the treatment with revulsant [3]. Therefore, to cover the complete picture of such process and pay attention to the secondary phase, we set the end time on the 20^th^ day rather than the 9^th^ day in the present study. After inhalation of acrolein fog for 20 days, marked mucus hypersecretion, substantial infiltration of inflammatory cells, serous effusion, and proliferation of alveolar epithelial cells were observed in airway and peribronchus tissues of mice. Additionally, total and neutrophilic cell counts in BALF were increased. Together with the hyperplasia of smooth muscle cells, all of these showed the typical pathological changes of airway remodeling, which was similar to the rat model established by Chen et al. in 2013 [30]. On the other hand, Masson stain revealed collagen deposition, airway interval thickening, and peribronchus fibrosis, which meant the fibrogenic progress and coincided with the representation of the secondary phase as expected. The expression of collagen protein was significantly increased during tissue repairing. This was in accordance with previous studies [31].

Hydroxyproline is a hydroxylated form of the proline, which is a kind of amino acid contained in the peptide chains forming collagen. Meanwhile, with the catalysis of collagenase, hydroxyproline is formed as a decomposition product of collagen. The process is essentially dynamic during fibrosis [32]. Therefore, we measured the hydroxyproline concentration of lung tissues to indirectly reflect the metabolic situation of collagen. Unexpected, there was no statistical difference in hydroxyproline concentration between each group on the 20^th^ day, which was quite different from the other PF models induced by bleomycin, asbestos, or paraquat. We considered this might be due to the unique physicochemical property of acrolein. Bleomycin, asbestos, and paraquat were more likely to induce acute tissue damage and lung fibrosis, while acrolein inclined the model to chronic progress. However, we did discover the collagen deposition and peribronchus fibrosis by Masson stain. As the secondary phase continued, hydroxyproline concentration of lung tissues might be increased, which needed further experiments to confirm.

Intervention in the process of airway remodeling at an early stage may contribute to regulating tissue repairing and fibrogenic progress, which would eventually cause physiological dysfunction of airway [33]. As Selroos et al. declared, early intervention with inhaled anti-inflammatory drugs in asthma might prevent patients from developing chronic airway obstruction [34]. The problem is in which joint we can break the chain. TGF-*β*1 plays an important role in cell growth, differentiation, and inflammation reaction. TGF-*β*1 could take effect in tissue repairing via promoting collagen synthesis [35]. In the previous studies, TGF-*β*1 was found to be involved in the MAPK, JNK, SMAD, and PI3K signaling pathways [36]. Recently, more and more researchers have begun to pay attention to the effect of TGF-*β*1 in the NF-*κ*B signaling pathway, especially in the animal models of tissue fibrosis. Chen et al. declared that through inactivation of NF-*κ*B but not the ERK1/2 signaling pathway, proliferation and migration of rat airway smooth muscle cells induced by TGF-*β*1 were inhibited [37]. In the same year, Zhao et al. also discovered that through the inhibition of NF-*κ*B signaling, proinflammatory and fibrogenic phenotypes of lipopolysaccharide-stimulated hepatic stellate cells were attenuated [23]. Researchers above used the CAPE as an inhibitor of NF-*κ*B in their study. In this study, CAPE attenuated the release of TGF-*β*1 and inhibited the fibrogenic progress in a model of airway remodeling induced by acrolein. In our study, we also identified the inhibitive effect of CAPE on NK-*κ*B pathway activation was related to the inhibition of P65 phosphorylation in mouse airway smooth muscle cell.

Muc5ac is a representative mucus protein, which is widely used as an evaluation criterion of airway secretion. The NF-*κ*B signaling pathway possibly takes part in such process. Now that CAPE, as an inhibitor of the NF-*κ*B pathway, took a protective effect on airway remodelling in our model, would it also play a role in prevention of Muc5ac overproduction and hypersecretion? Unfortunately, we observed obvious increases of Muc5ac mRNA level in lung tissue and Muc5ac protein level in BALF after being treated with acrolein. However, the increased levels of Muc5ac mRNA and muc5ac protein were not affected by the administration of CAPE. This suggested the inhibitions of airway mucin overproduction and hypersecretion were not the roles that CAPE played. This needs to be confirmed by further experimental studies.

In conclusion, CAPE, an inhibitor of the NF-*κ*B pathway, inhibited the process of acrolein-induced lung fibrosis in mice and attenuated the release of TGF-*β*1. This provides a theoretical basis for CAPE to be a clinical treatment for pulmonary fibrosis.

## Figures and Tables

**Figure 1:** Histopathological examination of lung tissue section by H&E staining. (a) Representative pictures of H&E staining. Scale bars = 200 *μ*m. Magnification: ×400. (b) Ashcroft Score for the image. CAPE: caffeic acid phenethyl ester. ^∗^*P* < 0.05 vs. the control group; ^#^*P* < 0.05 vs. the acrolein group.

**Figure 2:** Fibrosis examination of lung tissue by MASSON staining. Scale bars = 200 *μ*m. Magnification: ×400. Blue color indicates collagen deposition. CAPE: caffeic acid phenethyl ester.

**Figure 3:** Total and differential cell count in bronchoalveolar lavage (BALF). After inhalation of acrolein for 20 days, total cell count and neutrophilic granulocyte count were measured in BALF compared. CAPE: caffeic acid phenethyl ester. ^∗^*P* < 0.05 vs. the acrolein group.

**Figure 4:** Hydroxyproline concentration of lung tissues. Hydroxyproline concentration of lung tissue was detected by a hydroxyproline assay kit. CAPE: caffeic acid phenethyl ester.

**Figure 5:** TGF-*β*1 level in bronchoalveolar lavage (BALF). TGF-*β*1 level in BALF was detected by ELISA assay. CAPE: caffeic acid phenethyl ester. ^∗^*P* < 0.05 vs. the acrolein group.

**Figure 6:** Muc5ac level in lung tissue. (a) The protein expression of Muc5ac in the lung tissue was detected by Western blot. (b) The mRNA expression of Muc5ac in the lung tissue was detected by RT-qPCR. CAPE: caffeic acid phenethyl ester. ^∗^*P* < 0.05 vs. the control group.

**Figure 7:** Muc5ac protein level in bronchoalveolar lavage (BALF). The Muc5ac protein level in BALF was measured by ELISA. CAPE: caffeic acid phenethyl ester. ^∗^*P* < 0.05 vs. the control group.

**Figure 8:** P65 phosphorylation level in the TGF-*β*1-induced smooth muscle cells. (a) The protein expressions of phospho-P65 and P65 were detected by Western blot. (b) The ratio of p-P65/P65 was quantified. TGF-*β*1 group: the smooth muscle cells were treated with 10 ng/ml TGF-*β*1 for 30 minutes; TGF-*β*1+CAPE group: before stimulation with TGF-*β*1, the cell was pretreated with CAPE (100 nM) for 30 minutes. ^#^*P* < 0.05 vs. the control group. ^∗^*P* < 0.05 vs. the TGF-*β*1 group.

## Data Availability

The data used to support the findings of this study are available from the corresponding author upon request.
